# Stress Estimation Model for the Sustainable Health of Cancer Patients

**DOI:** 10.1155/2022/3336644

**Published:** 2022-07-25

**Authors:** Muhammad Adeel, Zahid Mehmood, Amin Ullah

**Affiliations:** ^1^Department of Computer Science, School of Science, National Textile University, Faisalabad 37610, Pakistan; ^2^Department of Computer Engineering, University of Engineering and Technology, Taxila 47050, Pakistan; ^3^Institute of Electrical Electronics and Computer Engineering, University of the Punjab, Lahore 54590, Pakistan

## Abstract

Good health is the most important and very necessary characteristic for stress-free, skillful, and hardworking people with a cooperative environment to create a sustainable society. Validating two algorithms, namely, sequential minimal optimization for regression (SMOreg) using vector machine and linear regression (LR) and using their predicted cancer patients' cases, this study presents a patient's stress estimation model (PSEM) to forecast their families' stress for patients' sustainable health and better care with early management by under-study cancer hospitals. The year-wise predictions (1998-2010) by LR and SMOreg are verified by comparing with observed values. The statistical difference between the predictions (2021-2030) by these models is analyzed using a statistical *t*-test. From the data of 217067 patients, patients' stress-impacting factors are extracted to be used in the proposed PSEM. By considering the total population of under-study areas and getting the predicted population (2021-2030) of each area, the proposed PSEM forecasts overall stress for expected cancer patients (2021-2030). Root mean square error (RMSE) (1076.15.46) for LR is less than RSME for SMOreg (1223.75); hence, LR remains better than SMOreg in forecasting (2011-2020). There is no significant statistical difference between values (2021-2030) predicted by LR and SMOreg (*p* value = 0.767 > 0.05). The average stress for a family member of a cancer patient is 72.71%. It is concluded that under-study areas face a minimum of 2.18% stress, on average 30.98% stress, and a maximum of 94.81% overall stress because of 179561 expected cancer patients of all major types from 2021 to 2030.

## 1. Introduction

There is an intense need for a sustainable society for every resilient city in the world, and this need is fulfilled by such people who have the characteristics which can play the role of pillars to develop a successful civilization. These characteristics include “unstressedness,” “skillfulness,” “hardworking,” and “cooperativeness.” Cancer is one of the most devastating diseases and causes many deaths. It was reported that, in 2020, from 185 countries, 19.3 million new cases of 35 types of cancer and 18.1 million cases of nonmelanoma skin cancer were estimated, whereas 10.0 million people died from 35 cancer types and 9.9 million patients died only from nonmelanoma skin cancer [1]. From 1998 to 2020, 201767 patients, with different cancer types, were registered within these 23 years only in three hospitals in the Punjab province of Pakistan. Therefore, cancer has become a great burden for sustainable public health. It has become the cause of immense stress for all family members if there is a cancer patient in the family. Such family members cannot work hard, even having qualities like “skillfulness,” “hardworking,” and “cooperativeness,” to create a sustainable society for a resilient city.

Machine learning gave us different algorithms to implement for social sciences in data mining [2–7]; mostly, regression models are used for prediction. Linear regression is implemented to predict the value for a dependent variable using independent values. Multiple regression uses several explanatory variables to predict the outcome of a response variable. Using a support vector machine (SVM) [8], sequential minimal optimization (SMO) [9] was proposed for solving the regression problem [10]. SMOreg was an improvement to SMO for SVM regression presented by Shevade et al. [11]. A study compared linear regression and SMOreg for predicting in the business area [12].

Good health is the most important and very necessary characteristic for stress-free, skillful, and hardworking people with a cooperative environment to create a sustainable society. As discussed above, cancer has become the cause of immense stress for all family members if there is a cancer patient in the family. Such family members cannot work hard, even having qualities like “skillfulness,” “hardworking,” and “cooperativeness,” to establish a viable civilization. Therefore, to overcome or reduce this stress on the families, there is a need for early management by every hospital for better care of cancer patients, especially in underdeveloped countries like Pakistan. This study presents a model to forecast their families' stress for patients' sustainable health and better care with early management by under-study cancer hospitals. To use the predicted number of new cases from 2021 to 2030 in the estimation of the stress, this study also validates the predicted results by linear regression and SMOreg, because some of the previous studies validated and others did not verify the forecasted cases of cancer patients.

## 2. Literature Review

Literature has intensive work regarding prediction models for different diseases. Reddy et al. presented an adaptive genetic algorithm with a fuzzy logic model to predict devastating heart disease with a better approach to predicting at early stages [13]. A study proposed a novel approach for classifying the infant cries of a newborn into three groups such as sleep, hunger, and discomfort [14]. Ramaneswaran et al. proposed a hybrid Inception model that is v3 XGBoost for the classification of severe and deadly disease, lymphoblastic leukemia, from microscopic images of white blood cells [15]. Gundluru et al. designed a model based on deep learning for dimensionality reduction with principal component analysis; an algorithm of Harris hawks optimization was also implemented for optimization of the classification and process of feature extraction. They also extracted the most important features in this regard [16]. The approach of structural equation modeling was used to study the relationships between mental health and parenting stress [17]. The approaches of structural equation modeling and confirmatory factor analysis were used to trial the posttraumatic growth role, physical growth, resilience, and mindfulness for the prediction of health-related and psychological adjustment [18]. Mediation analyses and multivariate regression were used for clarification of the extent to which coping strategies, psychological symptoms, and sleep quality with social support interfere as well as whether they arbitrated the relationship between fatigue or functional capacity and sleep quality in a sample of lung cancer patients treated with chemotherapy [19]. Stress patterns in connection with social support networks of hospice care were shared by Guo et al. [20]. Patient stress was classified with experiments from blood volume pulse by Lisowska et al. [21]. The stress level with related aspects in cancer patients was discussed by Durangi et al. [22]. Mikkelsen et al. shared the effect of emotional therapy in psychologically upset caregivers of tumor patients [23]. Stress in cancer patients was assessed by Safaei and Shokri using a factorial validity factor [24]. The research community has also published fruitful results regarding predictions for coming years to give oncologists better management and healthcare ideas during the treatment of this lethal disease [25–34]. A study presented a comprehensive analysis discussing the risk of incidence of subsequent hematological malignancies for primary tumors in cancerous patients [35]. The performances on the Wisconsin Breast Cancer dataset of different machine learning algorithms including Decision Tree, *k* Nearest Neighbors, support vector machine, and Naive Bayes were compared to observe the accuracy in classifying that dataset regarding the effectiveness and efficiency of each algorithm [32].  Table 1 shows the related results about developments in different areas published in recent years. In 2012, worldwide mortality and incidence rates of breast cancer were investigated using age-specific mortality and incidence rates [31]. Breast cancer statistics of four countries, including the US, UK, Egypt, and India, were shared in 2015 [26]. According to a prediction, around 3.2 million new cases of female breast cancer worldwide per year will be seen by 2050 [27].

## 3. Method

There are three parts of this study. The first part evaluates the used approaches (LR and SMOreg), and the second part forecasts and compares the number of predicted cases of cancer patients (by these approaches) to be used in the third part of the study, whereas the third part shows the proposed model (patient's stress estimation model) by this study.

### 3.1. Patients and Datasets

A total of 219882 cases of cancer patients registered from 1998 to 2020 were obtained with year-wise details from three sources. The first data source was the record room of the Clinical Oncology Department of Allied Hospital, Faisalabad Medical University, Faisalabad, Pakistan. The second data source of this study was Shaukat Khanum Cancer Registry [36] at Shaukat Khanum Memorial Cancer Hospital and Research Centre, Lahore, Pakistan, whereas the third source of the data, used in this study, was derived from a previous study [37]. After data cleaning and organization, cases of 2815 repeated incidences were removed, and finally, 217067 cancer patients were listed year-wise in two parts of the dataset for this study. The first part named, “CancerPatients1998to2010,” contained the cases of 88710 patients listed year-wise from 1998 to 2010. The second part named, “CancerPatients1998to2020,” had a list of 217067 patients saved year-wise from 1998 to 2020. The adopted methodology of this study is shown in Figure 1.

### 3.2. Configuration to Implement LR and SMOreg

#### 3.2.1. Configuration for Forecasting Cancer Patients from 2011 to 2020

The dataset, “CancerPatients1998to2010,” was used in the first part because we wanted to evaluate both approaches before forecasting new cancer incidences from 2021 to 2030. Therefore, in the first part, the LR model and SMOreg were implemented to predict the number of cancer patients from 2011 to 2020 providing a list of cancer patients registered from 1998 to 2010. LR and SMOreg were configured by five properties including “selected attribute,” “number of times units to forecast,” “timestamp,” “periodicity,” and “confidence interval” providing them with values “patients,” “10,” “year,” “yearly,” and “95%,” respectively.

#### 3.2.2. Configuration for Forecasting Cancer Patients from 2021 to 2030

In the second part, again, LR and SMOreg were implemented with the same configuration, as discussed in Section 3.1, to forecast the year-wise number of patients from 2021 to 2030 using the “CancerPatients1998to2020” dataset. Then, there was a need to compare the forecasted values by both approaches. The next section elaborates on the analysis methods used to compare the differences between the predicted values and the known values listed in the dataset.

### 3.3. Methods to Evaluate Predicted Values by LR and SMOreg

#### 3.3.1. Comparing the Predicted Incidences from 2011 to 2020 with the Known Cases

Based on a year-wise number of patients from 1998 to 2010, the predicted values (from 2011 to 2020) by LR and SMOreg were analyzed by getting their root mean square error (RMSE) to observed (actual) year-wise number of patients from 2011 to 2020. RMSE_1_ and RMSE_2_ for LR and SMOreg, respectively, according to values from the list in the “CancerPatients1998to2020” dataset, were then compared for the conclusion. The detail of this analysis is given in Statistical Analysis of this study.

#### 3.3.2. Comparing Predicted Incidences by Both Approaches from 2021 to 2030

Based on a year-wise number of patients from 1998 to 2020, the predicted values (from 2021 to 2030) by LR and SMO were analyzed by the statistical *t*-test. The detail of this analysis is given in Statistical Analysis.

### 3.4. Patient's Stress Estimation Model

In the third part of this study, a model, called patient's stress estimation model (PSEM), is proposed to estimate stress, faced by family members and society. PSEM is presented by using three categories of important factors (are discussed in Section 3.4.1) that play a major role in the implementation of PSEM. These factors were derived from the observations and interviews of the under-study patients' data. There are three equations derived for PSEM (Figure 2). The first equation uses two stress-impacting factors: (1) financial aspects and (2) affiliation, for PSEM to estimate stress for a family member of a cancer patient, and the second equation uses three other factors: (1) number of working family members of cancer patients, (2) number of dependent family members of cancer patients, and (3) number of expired cancer patients in a family, for PSEM to calculate total stress for a family of a cancer patient, whereas the third equation uses two factors: (1) number of families with cancer patient in the under-study areas and (2) population of the areas of under-study hospitals for PSEM to estimate overall stress for all cancer patients of the areas of the patients from under-study hospitals. The structure and working of PSEM (Figure 2) are explained in the following sections.

#### 3.4.1. Patient's Stress-Impacting Factor

There are deep relationships among people. These affiliations create an emotional linkage not only with their family members but also with their neighbors, colleagues, and friends. This link produces pleasure in them on other's success with good health. It also causes stress for them when they see a person in their relationship becomes a patient, especially a chronic patient. From the observation and interviews with the under-study patients and with their family members, it was derived that, when a person suffers from cancer, his or her family member becomes stressed because of two major reasons including affiliations and financial aspects. In affiliations, as the first stress-impacting factor, this study includes “father,” “mother,” “child,” “brother,” “sister,” “friend,” “colleague,” and “neighbor,” whereas “(is patient) working person,” “expired,” “physical status,” “income status,” and “treatment expenses” are financial aspects included by this study as the second stress-impacting factor. Other factors that take part in the calculation of total stress for a family of a cancer patient (s) are “number of working family members,” “number of independent family members,” and “number of expired patients in a family” included in this study.

#### 3.4.2. Estimating Stress for a Family Member of a Cancer Patient

The first equation of PSEM was derived by this study which is given below:

(1) $$\begin{array}{c} \text{Sf}=A+\left(\text{wP}\times E\right)+\left(\text{pS}\times \text{iS}\right)+eT, \end{array}$$

where Sf denotes the stress for a family member of a cancer patient. *A* is an affiliation that may be of five types including father/mother, child, brother/sister, friend, and colleague/neighbor. To estimate the stress, these types are assigned weights: 5, 4, 3, 2, and 1, respectively. wP is for getting input on the question: “Is the cancer patient working person?”; if the answer is “yes,” then wP is assigned 10 and 5 otherwise. *E* is for getting input on the question: “Is the cancer patient expired?”; if the answer is in “yes,” then *E* is assigned 7 and 4 otherwise. The variable pS is for getting input on the question: “What is the physical status of the cancer patient, can he/she work?” The answer may be “cannot work,” “can work 25%,” and “can work 50%” and is assigned weights: 5, 2, and 1, respectively. The variable iS is for getting input on the question: “What is the income status of the cancer patient?” The answer may be “cannot work,” “can work 25%,” and “can work 50%,” and is assigned weights: 5, 2, and 1, respectively. The variable eT is for the taking input of the question: “What are the expenses for treatment of the cancer patient?”. The answer may be “self,” if no funding was available; “self and free,” if some funding was available; and “free,” if funding was available. For “self” and “free,” 10 and 1 weights are assigned, respectively, whereas from 2 to 9, weights are assigned for self and free according to the available funding ratio to self-expenses on the treatment of the cancer patient. All the weights are assumed to get the values mathematically calculated. The observation of the under-study data and most of the interviews with many patients derived this study to suppose the above weights.

#### 3.4.3. Calculating Total Stress for a Family of a Cancer Patient

After estimation of stress for a family member of a cancer patient, PSEM is required to calculate total stress for the whole family of the cancer patient (s). Therefore, using Equation (1) and other factors including “number of working members of a family of a patient (s),” “number of dependent members (who do not work) of a family of a patient (s),” and “number of an expired cancer patient (s) in that family,” the following equation was derived by this study to calculate total stress for the whole family of a cancer patient (s) (Figure 2).

(2) $$\begin{array}{c} \text{TS}=\text{Sf}\times \left(\left|\text{nD}-\text{nW}\right|+1\right)+\text{nE}, \end{array}$$

where TS denotes the total stress for the whole family of a cancer patient (s). Sf is the stress for a family member of a cancer patient, calculated by Equation (1). nD is the number of dependent members (who do not work) of a family of a patient (s). nW is the number of working members of a family of a patient (s), whereas nE is the number of expired cancer patients in that family.

#### 3.4.4. Estimating the Overall Stress of All Cancer Patients in Under-Study Areas

Using Equations (1) and (2), PSEM derives the third equation (given below) to estimate overall stress for all cancer patients in the under-study areas.

(3) $$\begin{array}{c} \text{OES}=\left[\frac{\sum_{\text{nF}}\text{T}\text{S}}{\text{pA}}\right]\times 100 \end{array}$$

where OES denotes the overall estimated stress of all cancer patients in under-study areas. nF is the number of families with cancer patients in the under-study areas. TS is the total stress for the whole family of a cancer patient, calculated using Equation (2), whereas pA is the population of the areas of under-study hospitals. Suppose there are 35 families in the area with cancer patients, then the numerator of the given fraction will add the total stresses of 35 families, and then, this sum is divided by the population of that area.

## 4. Experimental Results

### 4.1. Evaluating and Validating the Predictions by LR and SMOreg

#### 4.1.1. Forecasting and Verifying the Incidences of Cancer Patients from 2011 to 2020

In the first part of this study, both LR and SMOreg were implemented to forecast for ten years the number of patients from 2011 to 2020 based on the year-wise known (observed) number of patients from 1998 to 2010. Linear regression and SMOreg predicted 117225 and 118644 patients, respectively, whereas 128357 patients were observed in these ten years (from 2011 to 2020) registered in the under-study hospitals in Punjab in Pakistan. LR predicted 10004, 9851, 10516, 11390, 11396, 11950, 12832, 13051, 13402, and 14253 number of cancer patients in the under-study hospitals from 2011 to 2020. SMOreg forecasted 10151, 10116, 10312, 11371, 11554, 11705, 12354, 13046, 13084, and 13533 cancer patients in the under-study hospitals from 2011 to 2020.

#### 4.1.2. Forecasting Year-Wise New Incidences of Cancer Patients from 2021 to 2030

In the second part of this study, both linear regression and SMOreg were implemented to forecast for ten years the number of patients from 2021 to 2030 based on the year-wise known (observed) number of patients from 1998 to 2020. Linear regression and SMOreg predicted 179561 and 181768 patients, respectively. LR predicted 3088, 3196, 3336, 3198, 3521, 3640, 3767, 3821, 3996, and 4117 number of expected cancer patients in the under-study hospitals from 2011 to 2030. SMOreg forecasted 3225, 3464, 3688, 3779, 3724, 4089, 4291, 4487, 4619, and 4737 expected cancer patients in the under-study hospitals from 2021 to 2030.

### 4.2. Statistical Analysis

There is a need to compare and evaluate the performance in forecasting the year-wise number of patients from 2011 to 2020 by LR and SMOreg. Therefore, their RMSE_1_ and RMSE_2_ are calculated that are 1076.15 and 1223.70, respectively, using the following equation [38]:

(4) $$\begin{array}{c} \text{RMSE}=\sqrt{\frac{\sum_{i=1}^{n}{\left(P_{i}-O_{i}\right)}^{2}}{n}}, \end{array}$$

where *P* denotes the predicted value, *O* is the observed value, and *n* is the number of forecasting instances, whereas *i* = 1, 2, 3, ⋯*n*. Analyzing the statistical difference between LR and SMOreg in forecasting the year-wise number of patients from 2021 to 2030, a *t*-test is applied. A two-sample *t*-test value of *N* applied for these models is 10. The means of the values predicted by LR and SMOreg are 17956 and 18177, standard deviations values are 1609 and 1667, and SE means values are 509 and 527, respectively. There is a -221 estimate for the difference, and a 95% confidence interval for the difference was (-1767, 1325). The *t*-value is -0.30, the *p* value is 0.767, and the value of the degree of freedom is 17.

### 4.3. The Estimated Stress for a Family Member of Cancer Patients

In the third part of the study, to forecast (2021-2030) overall stress for all expected cancer patients of the under-study areas using PSEM, there was a need to calculate TS, total stress, for a family of a cancer patient and thus, Sf was required to be calculated because it had been used in Equation (2). Sf is stress for a family member of a cancer patient (see Section 3.4.2). Therefore, it was observed that many patients had common values of patient stress affecting factors including *A*, wP, *E*, pS, iS, and eT (these variables have already been discussed in Section 3.4.2). Using Equation (1) with these common values, the calculated Sf is given in Table 2.

### 4.4. The Calculated Total Stress for a Family of a Cancer Patient

As discussed in Section 3.4.4, total stress for a family of a cancer patient, TS is required in the calculation of Equation (3). Therefore, it was observed that many patients had common values of nW, nD, and nE factors involved in the calculation of Equation (2) (these variables have already been discussed in Section 3.4.4). Using Equation (2) with these common values, the calculated TS is given in Table 3.

### 4.5. Overall Estimated Stress for Expected Cancer Patients of the Under-Study Areas

Finally, Equation (3) forecasted overall stress, from 2021 to 2030, for expected cancer patients of the under-study areas. Equation (3) used the total population of all under-study areas by getting the predicted population [39, 40] of each area from 2021 to 2030. OES calculation also needed nF, the number of families with possible cancer patients. Therefore, it used the predicted number of patients by linear regression, (see Section 3.2.2), since LR predictions are validated in Section 3.2.1. The overall stress (with average, minimum, and maximum value of TS) for expected cancer patients of the under-study areas forecasted (2021-2030) by using PSEM is given in Table 4.

## 5. Discussions

Part 1 of this study concludes that (based on the observed number of patients registered from 1998 to 2010 in the under-study hospitals) linear regression is better in forecasting the year-wise number of patients from 2011 to 2020 than that of SMOreg because RMSE_1_ (1076.15) is less than RMSE_2_ (1223.70). The statistical analysis of part 2 finds that there is no significant statistical difference between the year-wise number of patients from 2021 to 2030 predicted by linear regression and that of SMOreg because the *p* value (0.767) is not less than 0.05. The linear regression model predicts 179561 patients, whereas SMOreg predicted 181768 patients from 2021 to 2030. This is the reason for using the forecasted year-wise patients by LR from 2021 to 2030 because, as discussed already, linear regression is better in forecasting the year-wise number of patients from 2011 to 2020 than that of SMOreg. After all, RMSE_1_ (1076.15) is less than RMSE_2_ (1223.70). This study finds that linear regression performance remains better than that of SMOreg. Further, observing a total of 217067 already registered cancer patients from 1998 to 2020, it is estimated that the under-study hospitals will register 15493, 16119, 16658, 17183, 17707, 18231, 18755, 19280, 19805, and 20330 new cases of cancer patients from 2021 to 2030, respectively.

As discussed in “Method,” the third part of this study drives patients' stress-impacting factors and estimates stress for a family member of a cancer patient, total stress for a family of a cancer patient, and the overall stress of all cancer patients. Unfortunately, we could not find any paper that was exactly relevant to the major contributions of this study; however, some studies presented some parts of these contributions.  Table 5 compares their relevant work and the approach used in this study.

## 6. Conclusion

This study, for expected cancer patients of the under-study areas, forecasts (2021-2030) by using the proposed model, PSEM, estimating 30.98%, 2.18%, and 94.81% with 328.43, 23, and 1003 average, minimum, and maximum values of TS, respectively. Thus, under-study areas face a minimum of 2.18% stress, on average 30.98% stress, and a maximum of 94.81% overall stress because of 179561 expected cancer patients of all major types from 2021 to 2030. Therefore, these families remain unsuccessful to create a sustainable society due to the stress of their cancerous family members. This study recommends that PSEM can also be used to calculate and forecast stress for patients with other chronic diseases.

## Figures and Tables

**Figure 1:** Adopted methodology for modeling to forecast stress for the sustainable public health by comparing linear regression and SMOreg, based on data of 217067 cancer patients registered from 1998 to 2020 in three hospitals.

**Figure 2:** The structure and working of the patient's stress estimation model (PSEM).

**Table 1:** The summary of the related results published in recent years.

Publishing year	Objective	Approach	Results
2017 [17]	To study the relationships between mental health, parenting stress, and dyadic adjustment among first-time parents	Structural equation modeling	Showed the full intervention effect of mental health between dyadic adjustment and parenting stress. An analysis for multigroup observed that the paths did not vary across fathers and mothers.
2018 [18]	To examine the role of physical posttraumatic growth, posttraumatic growth, resilience, and mindfulness in the prediction of psychological and health-related adjustment	Confirmatory factor analysis and structural equation modeling	Forecasted quality of life and improvement of lower distress. The relationship between adjustment and resilience was noticed to be negotiated.
2019 [19]	To clear up the extent to which coping strategies, psychological symptoms, and social support interfere with good sleep quality and whether they arbitrate the relationship between fatigue and sleep quality or functional capacity of lung cancer patients.	Multivariate regression and mediation analyses	119 patients were enrolled, 58.2% of whom were found having a poor sleep because of cancer stress.
2020 [13]	To forecast heart disease which will help a physician in the diagnosis of heart disease at early stages	Rough sets and fuzzy rule-based classification with adaptive genetic algorithm	Main strengths of the presented model where it could efficiently tackle noisy data even on a huge number of attributes.
2021 [14]	To categorize the infant cries of a newborn into three groups such as hunger, discomfort, and sleep	Acoustic feature engineering and the variable selection using random forests	Showed a mean accuracy of around 91% for most situations, and this showed the capability of the suggested great gradient boosting-powered grouped-support-vector network in the classification of neonate cry. Also, the presented approach had a fast recognition rate of 27 seconds in the recognition of those emotional cries.
2021 [15]	To classify severe lymphoblastic leukemia from microscopic images of white blood cell	Image feature extractor and a classification head	Exhibited that using an XGBoost versus softmax classification head enhanced classification performance. Further, the attention map of the extracted features by Inception v3 for interpretation of the features learned by the presented model.
2022 [16]	To detect diabetic retinopathy at the early stages giving better results than other published approaches	Harris hawks optimization	The proposed model surpassed the other leading machine learning algorithms. However, training time was minimized. It was victimized to overfitting producing a negative impact on results when the original dataset was employed. The performance of the proposed approach had been improved even with an increased dataset size by two times.

**Table 2:** The estimated stress (with common values of patient's stress affecting factors) for a family member of a cancer patient from under-study hospitals.

Affiliation (*A*) father or mother = 5, child = 4, brother or sister = 3, friend = 2, colleague or neighbor = 1	Working person (wP) yes = 10, no = 5	Expired (*E*) yes = 7, no = 4	Physical status (pS) cannot work = 5, can work 25% = 2, can work 50% = 1	Income status (iS) poor = 3, average = 2, rich = 1	Expenses for treatment (eT) self = 10, free and self = >1 and <10, free = 1,	Stress for family member of a cancer patient (Sf)
5	10	7	5	3	10	100
4	10	7	5	3	10	99
3	10	7	5	3	10	98
2	10	7	5	3	10	97
1	10	7	5	3	10	96
5	5	7	5	3	10	65
5	10	4	5	3	10	70
5	10	7	2	3	10	91
5	10	7	1	3	10	88
5	10	7	5	2	10	95
5	10	7	5	1	10	90
5	10	7	5	3	7	97
5	10	7	5	3	6	96
5	10	7	5	3	5	95
5	10	7	5	3	4	94
5	10	7	5	3	2	92
5	10	7	5	3	1	91
4	5	7	5	3	10	64
3	5	7	5	3	10	63
1	5	7	5	3	10	61
5	5	4	5	3	9	49
5	5	4	5	3	8	48
5	5	4	5	3	7	47
5	5	4	5	3	6	46
5	5	4	5	3	5	45
5	5	4	5	3	2	42
5	5	4	5	3	1	41
5	5	4	5	2	10	45
1	5	4	1	1	1	23

**Table 3:** The calculated total stress for a family of under-study hospitals' cancer patients with common values of factors involved in the calculation.

Stress for a family member of a cancer patient (Sf)	Number of working family members of a cancer patient (nW)	Number of dependent family members of a cancer patient (nD)	Number of expired cancer patients in a family (nE)	Total stress for a family of a cancer patient (TS)
100	2	11	2	1002
99	2	5	1	397
98	1	3	1	295
97	1	4	0	388
96	2	7	0	576
65	2	8	1	456
70	1	4	1	281
91	1	3	1	274
88	1	3	1	265
95	0	4	1	476
90	0	6	1	631
97	1	5	1	486
96	3	7	1	481
95	2	6	1	476
94	1	3	0	282
93	1	5	1	466
92	1	4	1	369
91	1	3	0	273
64	0	5	1	385
63	1	2	0	126
61	1	2	0	122
49	3	4	0	98
48	1	2	0	96
47	1	6	0	282
46	1	5	1	231
45	1	3	0	135
44	0	7	1	353
42	1	2	0	84
41	5	1	0	205
45	1	2	2	92
23	1	1	0	23

**Table 4:** Overall stress for expected cancer patients of the under-study areas forecasted (2021-2030) by using PSEM (PSEM: patient's stress estimation model proposed by this study; TS: total stress for a family of a cancer patient).

Year	Forecasted total number of families with a cancer patient	Forecasted total population of under-study areas	Overall estimated stress with 328.43 (average) TS	Overall estimated stress with 23 (minimum) TS	Overall estimated stress with 1003 (maximum) TS
2021	15493	16637186	30.49	2.14	93.31
2022	16119	17166568	30.74	2.16	94.08
2023	16658	17690235	30.83	2.17	94.35
2024	17183	18207267	30.90	2.17	94.57
2025	17707	18718658	30.97	2.18	94.79
2026	18231	19226391	31.05	2.18	95.01
2027	18755	19733393	31.12	2.19	95.23
2028	19280	20242985	31.19	2.19	95.43
2029	19805	20758846	31.24	2.19	95.59
2030	20330	21283844	31.28	2.20	95.71

**Table 5:** Comparison of our approach with previous approaches.

Approach used by	Developed own model	Derivation of patients stress-impacting factors	Estimation of stress for a family member of a cancer patient	Calculation of total stress for a family of a cancer patient	Estimation of the overall stress of all cancer patients
Guo et al. [20]	✗	✗	✓	✗	✗
Karabulutlu [41]	✗	✓	✓	✗	✗
Golden-Kreutz et al. [42]	✓	✗	✗	✗	✓
Barre et al. [43]	✗	✗	✗	✗	✓
Northouse et al. [44]	✗	✗	✗	✓	✗
PSEM (this study)	✓	✓	✓	✓	✓

## Data Availability

The authors have used publicly available data to support the findings of this study that is included within the article.
